# Astaxanthin ameliorates prenatal LPS-exposed behavioral deficits and oxidative stress in adult offspring

**DOI:** 10.1186/s12868-016-0245-z

**Published:** 2016-02-08

**Authors:** Md. Mamun Al-Amin, Rabeya Sultana, Sharmin Sultana, Md. Mahbubur Rahman, Hasan Mahmud Reza

**Affiliations:** Department of Pharmaceutical Sciences, North South University, Plot 15, Block B, Bashundhara, Dhaka, 1229 Bangladesh; The Queensland Brain Institute, The University of Queensland, St. Lucia, Brisbane, QLD 4072 Australia

**Keywords:** Astaxanthin, Lipopolysaccharide, Depression, Anxiety, Oxidative stress

## Abstract

**Background:**

Prenatal maternal lipopolysaccharide (LPS) exposure leads to behavioral deficits such as depression, anxiety, and schizophrenia in the adult lives. LPS-exposure resulted in the production of cytokines and oxidative damage. On the contrary, astaxanthin is a carotenoid compound, showed neuroprotective properties via its antioxidant capacity. This study examines the effect of astaxanthin on the prenatal maternal LPS-induced postnatal behavioral deficit in mice.

**Results:**

We found that prenatal LPS-exposed mice showed extensive immobile phase in the tail suspension test, higher frequent head dipping in the hole-board test and greater hypolocomotion in the open field test. All these values were statistically significant (p < 0.05). In addition, a marked elevation of the level of lipid peroxidation, advanced protein oxidation product, nitric oxide, while a pronounced depletion of antioxidant enzymes (superoxide dismutase, catalase and glutathione) were observed in the adult offspring mice that were prenatally exposed to LPS. To the contrary, 6-weeks long treatment with astaxanthin significantly improved all behavioral deficits (p < 0.05) and diminished prenatal LPS-induced oxidative stress markers in the brain and liver.

**Conclusions:**

Taken together, these results suggest that prenatal maternal LPS-exposure leads to behavioral deficits in the adults, while astaxanthin ameliorates the behavioral deficits presumably via its antioxidant property.

## Background

Administration of lipopolysaccharide (LPS) into pregnant rodents strongly impaired innate immune responses [1] without the presence of infection [2]. LPS has been widely used in rodents during pregnancy to study behavioral deficits and histological irregularities in the adult offspring [3–6]. Prenatal maternal LPS challenge increases pro-inflammatory cytokines that cross the placental barrier and interfere with the early stages of brain development. The developmental abnormality is expressed in the behavioral level during the adult stage of life. Human epidemiological data suggests, early infections can produce mental disorders [7].

Prenatal LPS-induced maternal immune activation model has been used to develop animal model of depression [8], anxiety [9–11], impairment in learning and memory [12, 13], schizophrenia [14–16] and autism [17, 18]. In addition, prenatal LPS-exposure is linked with the development of long-term physiological complications in the offspring animals [19]. During gestational period, a specific time window is critical in inducing neurodevelopmental disorder and impaired behavioral deficits in the rodent’s offspring [6]. In this window, LPS-exposure leads to produce cytokines that crosses the placental barrier, which in turn interrupts the processes of fetal brain development [20]. Prenatal LPS-exposure has shown to enhance the level of nitric oxide (NO), lipid peroxidation and depleted the level of glutathione in the maternal liver, embryo, and placenta [21]. LPS-induced intrauterine fetal death and growth restriction are associated with higher lipid peroxidation and glutathione depletion in maternal liver, placenta, and fetal liver [22]. Cytokine independent reactive oxygen species (ROS) production has also been reported even within 40 min after LPS stimulation to human umbilical vein endothelial cells [23].

Based on the current data, it is hypothesized that prenatal LPS administration may contribute to adult behavioral dysfunction. It is also thought that ROS might play a significant role in the progression of such dysfunction. We assume that antioxidant like astaxanthin may scavenge oxidative stress in the brain to improve the impaired brain function. Therefore, this study investigates- (i) the effect of prenatal maternal LPS-exposed behavioral disorders and oxidative damage in the adult offspring and (ii) the effect of a potential antioxidant (astaxanthin) treatment in this prenatal LPS-exposed model.

Previous study used LPS at various dose range including small (120 µg/kg, i.p.) at GD 15–17 [24], moderate (300 µg/kg, i.p.) at GD 16–17 [12] to high (800 µg/kg, i.p.) at GD 15–17 [25] in mice model of behavioral deficit. In this study, moderate dose of LPS (300 µg/kg, body weight) was selected for *Swiss albino* mice. On the contrary, astaxanthin (AST) is a carotenoid antioxidant, having 100–500 times greater antioxidant capacity than α-tocopherol [26]. The BBB crossing ability of AST was evident, and possess neuroprotective properties [27] by the restoration of antioxidant enzymes such as, superoxide dismutase and glutathione peroxidase, and reduction of lipid peroxidation (MDA) [28], down-regulation of increased nuclear factor-kappaB (NF-_k_B), and expression of inflammatory cytokines [29]. Moreover, astaxanthin treatment improves depressive-like behavior by reducing the level of IL-6 and IL-β in the frontal cortex [30]. AST has shown a dose-dependent anti-inflammatory effect, by suppressing NO, and tumor necrosis factor- α (TNF-α) production, through directly blocking nitric oxide synthase enzyme activity. It is hypothesized that AST might be an effective antioxidant treatment of choice to improve LPS-exposed oxidative stress in adult lives.

## Methods

### Animals

Adult (age: 6 months) female (n = 12) *Swiss albino* mice (weight: 30 ± 2 g) were used for this experiment. Animals were housed in animal cage (Tecniplast, Italy) at 21 ± 2 °C room temperature, relative humidity 55 ± 5 % and 12-h light/dark cycle; and feed pellets and water ad libitum. Females with vaginal plug were designated as on embryonic day (ED) 0. The experimental procedure was reviewed and approved by the institutional ethical committee at the Department of Pharmaceutical Sciences, North South University (NSU/PHA/2014/133-046), Dhaka, Bangladesh. Animals were handled in accordance with the international principles guiding the usage and handling of experimental animals (United States National Institute for Health Publication, 1985). Behavioral and neuroendocrine parameters might be influenced by different estrous cycle phases [31]. Therefore, estrous cycle in female offspring was monitored before deciding the day for behavioral test.

### Animal grouping

Female pregnant mice were divided into two groups at ED 16 and ED 17. Control_saline group (n = 6) received intraperitoneal water for injection (100 µl) (Fig. 1) and experimental group (n = 6) received intraperitoneal LPS (*Escherichia coli*, Sigma-Aldrich, USA) at a dose of 300 µg/kg, body weight. Forty pups were selected for the postnatal experiments. On postnatal day 23 offspring were weaned and separated based on the gender. Offspring male animals were randomly selected and further grouped into four on postnatal day (PD) 90 as- (i) control_saline (n = 10), (ii) control_AST (n = 10), (iii) LPS (n = 10) and (iv) LPS_AST (n = 10).

**Fig. 1:** Grouping of the experimental animals. Effects of astaxanthin treatment on the adult mice prenatally exposed to either LPS or saline (control). *Swiss albino* mice were either treated withwater for injection (100 µl, saline, n = 6) or LPS (300 µg/kg, body weight) via intraperitoneal route at ED 16 and ED 17. Offspring male animals were randomly selected and further grouped into four on postnatal day (*PD*) 90 as- (i) control_saline (100 μl saline, n = 10), (ii) control_AST (astaxanthin, n = 10), (iii) LPS (100 μl saline,n = 10) and (iv) LPS_AST (astaxanthin,n = 10). The treatment was given for 6 weeks (PD 91–132). On PD 133 open field test was conducted followed by tail suspension and hole-board test. At the end of the behavioral test, animals were sacrificed to collect tissue

Control mice received either oral saline (100 μl) or oral astaxanthin (2 mg/kg, body weight; while LPS group was exposed to prenatal LPS and later received either oral saline (100 μl) or oral astaxanthin (2 mg/kg, body weight for 6 weeks). Behavioral test was conducted within 3 days (PD 133, 134 and 135) in the order of open field test followed by tail suspension and hole-board test. Within this period we have not seen any estrous cycle that may affect our behavioral results. Earlier, we decided to extend the treatment period (astaxanthin) if estrous cycle would appear. At the end of the behavioral test, animals were sacrificed to collect tissue.

### Preparation of astaxanthin and lipopolysaccharide

LPS (300 μg/kg) from *E. coli*, Sigma Aldrich, USA was dissolved in sterile water for injection [32] while water for injection (100 μL) was purchased from pharmacy shops. Astaxanthin powder was received as a gift from Pharma raw Bangladesh. AST was dissolved in distilled water at a concentration of 600 μg/ml and administered orally at a dose of 2 mg/kg body weight; [33] for 6 weeks starting from PD 91 to PD132.

## Behavioral test

### Open field test

The open field test device was made of plastic wood material following measurements described earlier [34]. The light source was a 35 w bulb suspended approximately 1 m above the apparatus for background lighting. Mice were carried to the testing room in their home cages and handled by the tails and were placed in the apparatus and allowed to explore the field for 20 min. After each trail, apparatus was cleaned using 70 % ethanol and allowed to dry. The exploration was recorded for later analysis by using a Logitech™ 4mp webcam. Video was analyzed manually using Smart™ V 3.0 video tracking software developed by PanLab. During the analysis, center zone and periphery zone were defined where center zone consists of 34.5 × 34.5 cm.

### Hole-boardtest

Hole-board test device box was constructed using plastic wood (length: 42 cm, width: 42 cm, height: 30 cm) containing twenty holes (4 cm diameter) in the floor. We considered gross exploratory behavior as the number of head dips into the holes (placing the head or snout into the holes in the floor). Video camera was installed to record the frequency and duration of each dipping. Locomotion-related behavior was scored as the number of rearings. The hole-board was cleaned between sessions.

### Tail suspension test

Tail suspension test (TST) was conducted according to the previous procedure described [35]. Briefly, each mouse was suspended by its tail using a clamp, 2 cm from the distal end, for 5 min in a gray plastic box (40 cm high, 30 cm wide, and 20 cm deep), with the head about above the floor (60 cm). Duration of immobility (defined as the absence of all movement except for those required for respiration) and mobility time were recorded (in seconds) for 5 min. Animals that climbed their tails during TST were excluded. Mobility was termed as hind leg movement, while immobility was defined as the absence of whole-body movement.

### Tissue processing

Brain and liver tissues were processed according to our previous method [36]. Mice were anesthetized with 0.1 ml of ketamine (50 mg/ml) and perfused through the heart with cold 0.9 % NaCl and phosphate buffered saline (PBS) to remove blood from the brain and liver tissue. The whole brain was immediately removed and kept in a petridish containing saline on ice. Cortex (100 mg) regions from the brain and liver (100 mg) tissues were collected to prepare 10 % (w/v) homogenate in sodium phosphate buffer (30 mmol/l, pH 7.0) using Ultra-Turrax T25 (USA) homogenizer. Homogenized tissue samples were sonicated at 5 s cycle for 150 s using an ultrasonic processor.

## Oxidative stress estimation

### Lipid peroxidation (MDA)

Lipid peroxidation was estimated colorimetrically measuring thiobarbituric acid reactive substances (TBARS) as described previously [37]. Briefly, tissue homogenate (0.1 ml +Tris–HCl buffer, pH 7.5) was treated with 2 ml of (1:1:1 ratio) TBA-TCA-HCl reagent (thiobarbituric acid 0.37 %, 0.25 N HCl and 15 % TCA) and placed in water bath for 30 min and cooled. The absorbance of clear supernatant was measured against reference blank at 535 nm.

### Catalase (CAT)

Activity of catalase (CAT) enzyme was assayed at 240 nm and expressed as activity in percentage of H_2_O_2_ consumed/min/mg protein as described [38]. The reaction mixture (1.5 ml) contained phosphate buffer (1.0 ml) (0.01 M, pH 7.0), tissue homogenate (0.1 ml supernatant) and H_2_O_2_ (0.4 ml) (2 M). The reaction was stopped by the addition of 2.0 ml of dichromate-acetic acid reagent (5 % potassium dichromate and glacial acetic acid were mixed in 1:3 ratio).

### Nitric oxide (NO)

Nitric oxide was determined according to the method described by Tracy et al. as nitrate and nitrite [39]. NO level was measured by using standard curve and expressed as nmol/gm of tissue. Griess-Illosvoy reagent was modified by using naphthyl ethylene diaminedihydrochloride (NED) (0.1 % w/v) instead of 1-napthylamine (5 %). The reaction mixture (3 ml) containing brain homogenates (0.5 ml), phosphate buffer saline (0.5 ml), NED (1 ml) and sulfanilamide (1 ml) was incubated at 25 °C for 15 min. A pink chromophore was formed in diffused light. The absorbance of the solution was measured at 540 nm against the corresponding blank solution.

### Advanced protein oxidation product (APOP)

Advanced protein oxidation product was assayed based on spectrophotometric detection according to [40]. APOPs were expressed in chloramine units (nmol/ml). Briefly, plasma (50 µl diluted with phosphate-buffered saline (PBS) (100 µl), and chloramin T (0–100 mmol/l) were used for the preparation of calibration curve and PBS was used as blank. Potassium iodide (100 µl of 1.16 M) and acetic acid (50 µl) were added to each well and absorbance was taken at 340 nm immediately.

### Superoxide dismutase (SOD)

The activity of superoxide dismutase enzyme was assayed by a modified procedure described previously [41]. Briefly, each 300 μl reaction mixture contained 50 mM sodium phosphate (pH 7.8), 13 mM methionine, 75 mM nitrobluetetrazolium (NBT), 2 mM riboflavin, 100 mM EDTA, and 2 ml of plasma. The change of absorbance in each sample was then recorded at 560 nm after the production of blue formazan.

### Glutathione (GSH)

Glutathione in the brain was assayed according to the previous method [42]. Briefly, 1 ml of plasma was added with 2.7 ml of phosphate buffer (0.1 mol/l, pH 8) and 0.2 ml of 5, 5-dithio-bis (2-nitrobenzoic acid). The color developed was measured immediately at 412 nm. Results are expressed as μmol/mg protein.

### Statistics

The data of this present study was analyzed by one-way ANOVA to compare the main effect of astaxanthin on dependent variables in control_saline, control_AST, LPS, and LPS_AST groups. Post-hoc test namely “Newman-Keuls” was used as a multiple comparisons test to compare between groups. All analyses were carried out using GraphPad Prism software (version 6.0). The differences were considered significant when p values were at least less than 0.05. Data are represented as mean ± SEM (standard error of the mean).

## Results

### Behavioral studies

#### Open field test

A significant main effect of treatment on the number of entry into the periphery [F_(3,36)_ = 6.34, p < 0.01] (Fig. 2a), time spent in periphery [F_(3,33)_ = 6.95, p < 0.001] (Fig. 2b) and total distance travelled [F_(3,34)_ = 4.49, p < 0.01] (Fig. 2c) was observed for four conditions (control_saline, LPS, LPS_AST, control_AST). Neuman-keuls multiple comparison test showed that control_saline (M = 29.50, SD = 10.33), LPS_AST (M = 32.70, SD = 15.09) and control_AST (M = 44.50, SD = 18.45) groups had lower entry frequency in the periphery than LPS group (M = 63.10, SD = 27.99). Similarly LPS group (M = 949, SD = 147) spent longer time in periphery than control_saline (M = 695, SD = 167), LPS_AST (M = 804, SD = 141) and control_AST (M = 678, SD = 126) groups. Moreover, LPS group (M = 213, SD = 46) travelled lower distance than control_saline (M = 320, SD = 96), LPS_AST (M = 328, SD = 36) and control_AST (M = 301, SD = 133) groups.

**Fig. 2:** Effects of astaxanthin on locomotor activity in the open field test (*OFT*).The parameters of interest in the open field test are number of entry in periphery (**a**); time spent in periphery (**b**); and total distance travelled (**c**).Results were shown as mean ± SEM. *p < 0.05, **p < 0.01

#### Tail suspension test

There was a significant main effect of treatment on the duration of immobile time [F_(3,34)_ = 7.39, p < 0.001], and mobile time [F_(3,35)_ = 4.17, p < 0.01] for the four conditions (control_saline, LPS, LPS_AST, control_AST). Neurman-keuls multiple comparison test showed that control_saline (M = 179, SD = 47), LPS_AST (M = 172, SD = 67) and control_AST (M = 219, SD = 47) groups had lower immobile phase than LPS group (M = 269, SD = 39) (Fig. 3a). Likewise, control_saline (M = 167, SD = 43) and LPS_AST (M = 154, SD = 66) spent less mobile phase than LPS group (M = 91, SD = 39) (Fig. 3b). However, control_AST (M = 125, SD = 52) group did not show significant difference from any other groups.

**Fig. 3:** Effects of astaxanthin on immobility and mobility time in the tail suspension test (*TST*) and hole-board test in LPS-exposed mice. Results are shown as mean ± SEM. *p < 0.05, **p < 0.01, ***p < 0.001. Tail suspension test parameters are duration of immobility time (**a**) and duration of mobility time (**b**) while hole-board test parameters are frequency (**c**) and duration of head dipping (**d**)

#### Hole-board test

There was a significant main effect of head dipping frequency [F_(3,34)_ = 8.69, p < 0.001] (Fig. 3c) and head dipping duration [F_(3,36)_ = 9.86, p < 0.001] (Fig. 3d). Neurman-keuls multiple comparison test showed that control_saline (M = 43.0, SD = 6.5), LPS_AST (M = 46.3, SD = 4.3) and control_AST (M = 52.6, SD = 8.1) groups had lower frequency of head dipping than LPS group (M = 65.0, SD = 16.8). Additionally, control_saline (M = 81.8, SD = 27.2), LPS_AST (M = 76.7, SD = 20.1) and control_AST (M = 84.4, SD = 18.6) groups spent lower duration of head dipping than LPS group (M = 125.0, SD = 22.6).

#### Oxidative stress

One-way ANOVA analysis showed a significant main effect of treatment on the MDA level in brain [F_(3,36)_ = 6.19, p < 0.01] (Fig. 4a), and liver [F_(3,35)_ = 4.37, p < 0.01] (Fig. 4b); AOPP in the brain [F_(3,34)_ = 5.27, p = 0.01] (Fig. 4c), and liver [F_(3,34)_ = 18.06, p = 0.001] (Fig. 4d); NO in the brain [F_(3,33)_ = 40.47, p < 0.001] (Fig. 4e) and liver [F_(3,31)_ = 28.39, p < 0.001] (Fig. 4f); glutathione in the brain [F_(3,36)_ = 266.1, p < 0.001] (Fig. 4g) and liver [F_(3,35)_ = 16.79, p < 0.001] (Fig. 4h); catalase activity in the brain [F_(3,34)_ = 9.45, p < 0.001] (Fig. 4i) and liver [F_(3,36)_ = 16.27, p < 0.001] (Fig. 4j); and SOD activity in the brain [F_(3,34)_ = 6.97, p < 0.001] (Fig. 4k) and liver [F_(3,32)_ = 9.75, p < 0.001] (Fig. 4l) among the four treatment groups.

**Fig. 4:** Effects of astaxanthin on the oxidative markers in the brain and liver in prenatally LPS-exposed animals. Oxidative stress parameters are lipid peroxidation (*MDA*) in the brain (**a**) and liver (**b**); advanced oxidation of protein products (*AOPP*) in the brain (**c**) and liver (**d**); nitric oxide (*NO*) in the brain (**e**) and liver (**f**); glutathione (*GSH*) in the brain (**g**) and liver (**h**); catalase (*CAT*) in the brain (**i**) and liver (**j**); and superoxide dismutase (*SOD*) in the brain (**k**) and liver (**l**). Results are shown as mean ± SEM. *p < 0.05, **p < 0.01, ***p < 0.001

Neurman-keuls multiple comparison test indicated a lower level of MDA in the control_saline (M = 27.0, SD = 8.5), LPS_AST (M = 32.7, SD = 8.3) and control_AST (M = 29.5, SD = 4.3) groups than LPS (M = 40.7, SD = 8.7) in the brain. Similar findings were observed in liver MDA also. Likewise, lower level of AOPP was found in control_saline (M = 80.0, SD = 25.0), LPS_AST (M = 82.1, SD = 26.1) and control_AST (M = 40.3, SD = 3.5) than LPS (M = 121.6, SD = 12.3) in the brain. Similar findings were again observed in liver AOPP. In addition, control_saline (M = 3.2, SD = 2.1), LPS_AST (M = 8.3, SD = 1.9) and control_AST (M = 2.4, SD = 1.6) groups had lower NO than LPS (M = 11.2, SD = 2.2) in the brain. Similar results were observed in liver NO as well.

To the contrary, control_saline (M = 11.7, SD = 1.7), LPS_AST (M = 3.5, SD = 0.5) and control_AST (M = 16.2, SD = 1.7) groups had higher GSH than LPS (M = 1.2, SD = 0.6) in the brain. Interestingly, data from liver showed different result. Control_saline (M = 4.0, SD = 0.8) and LPS_AST (M = 3.2, SD = 1.0) had higher GSH than LPS (M = 2.2, SD = 0.5) and control_AST (M = 1.6, SD = 0.2). The level of CAT in the control_saline (M = 12.3, SD = 3.6), LPS_AST (M = 11.9, SD = 4.1) and control_AST (M = 16.4, SD = 1.5) was higher than LPS (M = 8.3, SD = 2.3) in the brain. Similar findings were further observed in liver CAT. SOD data revealed that control_saline (M = 21.4, SD = 6.5), LPS_AST (M = 21.5, SD = 5.9) and control_AST (M = 25.0, SD = 2.7) groups had higher SOD than LPS (M = 14.4, SD = 2.6) in the brain. Liver SOD levels were similarly consistent with that of the brain.

## Discussion

The result of the present study demonstrated that; prenatal LPS-exposure leads to anxiety and depressive like behaviors, and oxidative damage in the brain and liver during the adult lives. To the contrary, postnatal treatment with astaxanthin ameliorates impaired behavior and oxidative markers in the prenatal LPS-exposed offspring mice.

It has been demonstrated that prenatal maternal immune activation with LPS elicits behavioral deficits such as reduced locomotoractivity [9, 43] and social exploration [44] in the open field test in the adult lives [9]. In this study, prenatal maternal LPS-exposed animals have shown an increased time in the peripheral region and reduced global activity in the open field test. In addition, prenatal LPS-exposed animals have spent an increased immobility and reduced mobility time in the tail suspension test in the offspring. These indicate the development of behavioral deficits in the adult offspring of LPS group. Increased duration of immobility in the tail suspension test was also observed in the prenatally stressed rats [45] and mice [46]. To be noted that, when astaxanthin was given to healthy animals, it further showed similar effects as produced by prenatal LPS. This may be explained as the adverse effect of any potent drug/chemical when given at normal physiology. When the immunity was challenged by prenatal LPS, the therapeutic effect of astaxanthin became noticeable. It is important to note that, 6-weeks-long treatment with astaxanthin improves the parameters of open field and tail suspension test in the offspring animals. Ying et al. (2015) has shown that 10 weeks treatment with astaxanthin (25 mg/kg/day, body weight) increases locomotor activity by enhancing total travelling distance in the open field test [30].

Our results demonstrated that prenatal maternal LPS exposure leads to increased anxiety in the adult offspring as evident in the hole-board test. Our results are consistent with previous studies demonstrating that prenatal LPS-exposure in the late gestational stage resulted in increased anxiety and depressed behaviors in the adult mice. Prenatal LPS-exposed mice exhibited a higher level of anxiety as evident even in the postnatal day 240 [47]. To the contrary, treatment with astaxanthin reverses anxiety-like disorder in the mice. Our results are in line with the other studies [48, 49].

Our results depict that prenatally LPS-exposed animals had decreased levels of antioxidant enzymes such as, superoxide dismutase, catalase and glutathione, while an increased level of lipid peroxidation, protein oxidation products, and NO in the adult lives. These results indicated the correlation of prenatal administration of LPS with the oxidative stress in the adult lives. The depletion of antioxidant enzymes have shown by the other studies. For example, LPS-induced depletion of endogenous antioxidant enzymes including superoxide dismutase, catalase has been reported earlier [50].

LPS-induced lipid peroxidation has been shown in in vitro [51–53] and in vivo [54] animal studies. It has been revealed that LPS-exposure results in neurotoxicity via microglial activation. In-utero LPS-induction causes the activation of microglia. This activated microglia produces increased level of NO, ROS, and inflammatory cytokines such as TNF-α [55]. Activated microglia and astrocyte cells accelerate iNOS induction which results in the production of ROS. NO may harm oligodendrocytes and myelin which in turn interferes mitochondrial electron transport chain and translocates apoptosis inducing factor [56]. Thereby, oxidative stress may play a vital role in damaging axons via disrupting mitochondrial function. As a result, energy production will be dropped, protein and lipid would be oxidized, microtubule would be degraded, and axonal transport will be interrupted [57]. A recent study reports that axonal damage could be elicited by LPS-mediated microglia activation as well as by H_2_O_2_-promoted oxidative stress [58].

Prenatal LPS-exposure may lead to the brain damage due to the production of toxic free radicals (.OH) [59], and an increased level of superoxide anion (O2−) in the liver [60]. Free radicals react with the important biological substrates, including DNA, proteins, and lipids, which interrupt cell function and may lead to cell death. It has been reported that LPS induces the activation of microglia [61], reactive astrocyte [62], apoptosis of oligodendrocyte precursors which produces superoxide anion (O2−), and NO and contributes in neurodegeneration [63]. Moreover, LPS treatment triggered the production of ROS which in turn causes neuronal cell death in cortex and hippocampus [64, 65] and loss of dopaminergic neurons in the striatum [66]. ROS causes cellular damage including lipid peroxidation, interrupts the fluidity of membrane. Our result showed an increased MDA level in the prenatal LPS-exposed offspring brain and liver, which is consistent with the previous study [67].The level of glutathione was dropped in the prenatal LPS-exposed offspring. It is possible because of the action of glutathione against lipid peroxidation since it is responsible to reduce the level of peroxidized phospholipids and cholesterols [68]. Thus, the level of glutathione reserves could be depleted during oxidative stress as we observed in the prenatal LPS-exposure group.

Despite the LPS-induced oxidative damage, our results showed an improvement of oxidative markers after the treatment with astaxanthin in the adult lives. This study measured the concentration of MDA, NO, APOP, GSH and antioxidant enzyme activity (SOD and CAT) in the brain and liver). AST reduces prenatal LPS-induced elevated level of MDA, NO, APOP production and restores the concentration of GSH in the brain and liver. In-vitro studies were conducted to measure the effect of AST on LPS-induced oxidative stress in U937 [53] and RAW264.7 [69] cell line. Restoration of antioxidant enzyme activity (SOD and CAT) and inhibition of NO production have been shown by astaxanthin in such oxidative stress cell line. In addition, astaxanthin is believed to reduce inflammatory cytokine by its antioxidant property. It possibly inhibits elevated level of pro-inflammatory cytokines by blocking NF-kBactivation [69]. Ohgami et al. (2003) investigated the effect of AST on LPS-induced inflammation in in vitro and in vivo model. The author demonstrated that AST reduces the elevated NO production and prostaglandin E2 (PGE2) and TNF-α level where L-NAME was used as a positive control. The authors further suggest that reduction of NO production was due to the blocking of NOS enzyme activity similar to the NOS inhibitor L-NAME [70]. NO level was decreased with the treatment of astaxanthin. NO is involved as a neurotransmitter in the CNS which plays an important role in learning and memory. Previous study suggests that NO is released only during training [71]. Role of AST on NO (neurotransmitter) can be investigated during learning session. Since we did not measure the level of NO during training therefore, this result could not explain the effect of AST on signal transmission. However, the reduction of NO that is related with free radical induction is beneficial since neuroprotection is evident in the hippocampus by low level of lipid peroxidation and increased catalase activity.

The AST treatment was given for 6 weeks; from postnatal day 91 to 132 with the intent to reduce the stress level that was enhanced by prenatal LPS exposure in our mice model. This timing of AST treatment was rationally decided after reviewing the previous studies demonstrating neurochemical abnormalities in the adults after prenatal LPS administration [72–74]. In control_AST group, only astaxanthin was given to the animals that were not prenatally LPS-exposed for better comparison and to understand the effect of AST on prenatally LPS-exposed mice. Most of the parameters obtained from the behavioral test (except mobile phase duration in the tail suspension test) and oxidative stress markers were significantly improved in the brain and liver of the control_AST and LPS_ASTgroup. Only the GSH in the liver was not improved by astaxanthin as compared with LPS_AST group, which may be due to improper handling of tissue samples since our previous study as well as several other studies demonstrated a positive effect of AST on GSH in the liver [49, 75–77]. Newman-keuls post hoc test was done to determine the difference between the groups.

The result of the present study showed that astaxanthin treatment reduces a prominent marker of lipid peroxidation (MDA) which is also observed in the ischemic brain injury in adult rats [78]. Wu et al. investigated the protective effect of astaxanthin on D-galactose induced brain aging in rats. The authors demonstrated that astaxanthin treatment restored the activity of SOD, and increased GSH, which is in agreement with our present findings [28]. However, our study has several limitations; we were unable to conduct histology, proteomics, determination of cytokines and neurotransmitter because of lack resources and financial support in our lab. In addition, astaxanthin was given at a single-dose (2 mg/kg) for 6-weeks. Higher or lower dose of astaxanthin could be given to investigate the pharmacological profile of this antioxidant in animal model. Future study may include the determination of the aforesaid compounds to drill down more on the activity of astaxanthin on such prenatal maternal immune activated postnatal behavioral deficits model.

Nevertheless, the present study is novel in many respects. This study first addresses the effect of astaxanthinon the prenatal LPS-exposed behavioral disorder in the adult offspring in in vivo model. This study focused on the determination of six oxidative markers. The results of this study open a new avenue to explore the molecular mechanism of antioxidant (AST) in developing behavioral disorders. A further study with co-administration of astaxanthin and LPS in the prenatal stage to observe the protective effect of astaxanthin in the postnatal stage can be initiated.

## Conclusions

Prenatally LPS-challenged mice developed behavioral deficits such as depressive and anxiety like symptoms in the adult lives. However, treatment with a potential carotenoid antioxidant astaxanthin in the adult life for a period of 6 weeks showed a significant improvement in the behavioral disorders. We report that astaxanthin treatment possibly benefit depressive and anxiety episodes by reducing oxidative stress. This study thus predicts the potential of astaxanthin in the treatment of neuro-psychiatric disease, but future study should be conducted to explore underpinning mechanisms to ensure the findings.
